# The Recognition Method of Athlete Exercise Intensity Based on ECG and PCG

**DOI:** 10.1155/2022/5741787

**Published:** 2022-05-30

**Authors:** Baiyang Wang, Haiyan Zhu

**Affiliations:** Linyi University, Linyi, China

## Abstract

Athletes usually arrange their training plans and determine their training intensity according to the coach's experience and simple physical indicators such as heart rate during exercise. However, the accuracy of this method is poor, and the training plan and exercise intensity arranged according to this method can easily cause physical damage, or the training cannot meet the actual needs. Therefore, in order to realize the reasonable arrangement and monitoring of athletes' training, a method of human exercise intensity recognition based on ECG (electrocardiogram) and PCG (Phonocardiogram) is proposed. First, the ECG and PCG signals are fused into a two-dimensional image, and the dataset is marked and divided according to the different motion intensities. Then, the training set is trained with a CNN (convolutional neural network) to obtain the prediction model of the neural network. Finally, the neural network model is used to identify the ECG and PCG signals to judge the exercise intensity of the athlete, so as to adjust the training plan according to the exercise intensity. The recognition accuracy of the model on the dataset can reach 95.68%. Compared with the use of heart rate to detect the physical state during exercise, ECG records the total potential changes in the process of depolarization and repolarization of the heart, and PCG records the waveform of the beating sound of the heart, which contains richer feature information. Combined with the CNN method, the athlete's exercise intensity prediction model constructed by extracting the features of the athlete's ECG and PCG signals realizes the real-time monitoring of the athlete's exercise intensity and has high accuracy and generalization ability.

## 1. Introduction

Reasonable physical activity is good for health. However, it is easy to cause physical damage, tachycardia, and myocardial strain and ultimately life-threatening due to unreasonable high-intensity exercise methods. Athletes need to continuously improve their competitive ability, which requires higher-intensity physical training to tap their potential and achieve better results. Only by arranging training plans reasonably can physical injuries caused by excessive training intensity be prevented [1, 2].

In general, system indicators such as respiratory rate and heart rate are used to judge exercise intensity. These signals contain less information and cannot accurately and comprehensively reflect the state of exercise. Therefore, many researchers began to explore the use of other physical indicators that contain more information to evaluate physical status [3–6]. Kulawiec et al. [7] observed the blood glucose levels of athletes after exercise to judge recovery of athletes. Pero et al. [8] monitored various biochemical parameters including pH, leukocytes, red blood cells, protein, and glucose in urine after exercise, and based on these biochemical parameters, each athlete was provided with personalized treatment to monitor the athlete's health status. Wang and Yin [9] proposed the use of machine learning to monitor the physiological indicators of athletes, in which they use physiological indicators such as heart rate, maximum oxygen uptake, oxygen pulse, respiratory entropy, and maximum ventilation times and achieved good results. Compared with a single index to judge the motion state, the accuracy of these methods has been greatly improved. However, it is difficult to measure and judge in real time due to the limitations of the measuring instruments. Therefore, how to improve real-time monitoring is a major problem in exercise monitoring.

With the emergence of wearable devices and the miniaturization of monitoring devices, researchers have proposed different real-time monitoring systems to obtain more real-time heart rate information and related information [10–17]. Manas et al. [18] developed an intelligent, noninvasive wearable physiological parameter monitoring device that uses several different sensors to monitor human body temperature and heart rate and uses wireless networks to track human health status. Lei et al. [19] used support vector machines and multichannel PCG signals to build a model for measuring athletes' heart rate detection. Sujadevi et al. used a 3-layer CNN to detect PCG anomalies, and the resulting model achieved 80% accuracy.

In these studies, PCG and ECG are rich in features and have achieved high accuracy in different applications. In addition, PCG and ECG monitoring equipment has good portability and is more suitable for daily sports training [20–29]. Therefore, this study proposes a human exercise intensity recognition method based on ECG and PCG. In order to improve the monitoring accuracy, PCG and ECG signals are fused to monitor exercise intensity.

Heart rate, as a scalar, contains less information than methods such as heart rate extraction from PCG and ECG signals. For a specific sport, heart rate does not effectively utilize the information in the athlete's ECG and PCG. In this study, the complete PCG and ECG waveforms of a certain state are used as indicators, and the data are processed in two dimensions to identify, which will be more targeted. The deep learning method can also be personalized for a certain sport of an athlete and quickly establish a sports state model, so as to monitor the training more effectively. The direct use of PCG and ECG waveforms for classification and identification is more conducive to the accuracy of identification, and it has broad application prospects not only in identifying the current exercise intensity but also in disease prevention. The rest of the paper is organized as follows: Section 2 describes how to fuse the PCG and ECG signals together and convert the fused data into a dataset suitable for training a CNN, as well as the CNN network used to train the model. A Simultaneous Electrocardiogram and Phonocardiogram Database used in this paper is introduced in Section 3.  Section 4 presents the experimental procedure and results and discusses the results.  Section 5 gives the conclusion.

## 2. Methods

This section will briefly introduce the proposed athlete exercise intensity identification method based on ECG and PCG, which includes the AlexNet CNN structure and the fusion processing of ECG and PCG multisource signals. The method is validated using an open dataset from the Physical Web, which demonstrates that the use of ECG and PCG information can effectively discriminate the exercise intensity of athletes. In the rest of this section, the CNN, the model evaluation metrics, and the overall method flow will be described in detail.

### 2.1. AlexNet Network

This paper will use the AlexNet network proposed by Alex et al. The AlexNet network is a convolutional neural network with 5 convolutional layers, 3 pooling layers, and 3 fully connected layers designed by Hinton, the winner of the 2012 ImageNet competition, and his student Alex Krizhevsky [30]. AlexNet deepens the structure of the neural network on the basis of LeNet and uses stacked convolutional layers. Dropout is used to randomly ignore some neurons during training to avoid model overfitting. The ReLU function is used as the activation function, and CUDA (Compute Unified Device Architecture) is used to speed up the depth. And the parallel computing power of GPU is used to handle a large number of matrix operations during neural network training. The structure of AlexNet is shown in Figure 1.

### 2.2. Evaluation Indicators

#### 2.2.1. Loss and Accuracy Function

The advantages and disadvantages of the CNN model are usually measured by loss function and accuracy. Loss function is used to evaluate the difference between the predicted value and the real value of the model. The better the loss function is, the better the performance of the model is generally. The loss function used by different models is generally different. The cross-entropy loss function is used in this study. The cross-entropy is used to measure the distance between two different direction vectors and is a widely used loss function in multiclassification problems. The calculation formula is shown as Formula (1), where *n* represents the total number of samples and *m* is the number of categories. *y*_*ic*_ symbol function (0 or 1), if the true class of sample *i* is equal to *c*, take 1; otherwise, take 0. *p*_*ic*_ observes the predicted probability of sample *i* for category *c*:

(1) $$\begin{array}{c} \text{Loss}=\frac{1}{n}\underset{i}{\sum }\overset{m}{\underset{c=1}{\sum }}y_{ic}\log\left(p_{ic}\right). \end{array}$$

The accuracy evaluation index is the proportion of correct results obtained by classification in the total number of training models in a given test set. In classification, if one category is defined as positive, the other categories are negative. TP is the number of positive categories predicted to be positive; FP is the number of negative categories predicted to be positive; TN is the number of negative categories predicted to be negative; FN is the number of positive categories predicted to be negative. The definition of indicators is shown in

(2) $$\begin{array}{c} \text{Accuracy}=\frac{\text{TP}+\text{TN}}{\text{TP}+\text{TN}+\text{FP}+\text{FN}}. \end{array}$$

#### 2.2.2. Confusion Matrix

The confusion matrix is used to put the predicted results of all categories and the real results into the same table by category, and there are the number of correct identifications and the number of incorrect identifications for each category in this table. Taking Figure 2 as an example, there are two categories: 0 and 1. The diagonal line in the table is the number of correct identifications, TP is the number of positive categories predicted as positive, FP is the number of negative categories predicted to be positive, TN is the number of negative categories predicted to be negative class, and FN is the number of positive categories predicted as negative class.

#### 2.2.3. *t*-SEN (*t*-Distributed Stochastic Neighbor Embedding) Cluster Analysis

Cluster analysis of data can better observe the experimental results, find out the relationship between various categories, and make the data concise; thus, we can judge the quality of the training results more intuitively.

*t*-SNE is a machine learning algorithm for dimensionality reduction, which was proposed by Laurens van der Maaten and Geoffrey Hinton in 2008. *t*-SNE is a nonlinear dimensionality reduction algorithm. *t*-SNE technology can reduce the high-dimensional data of the fully connected layer of CNN to two-dimensional, so that we can visually and intuitively judge the performance of the current model [31].

### 2.3. CUDA (Compute Unified Device Architecture) Accelerated Processing

CUDA is a general-purpose parallel computing architecture introduced by NVIDIA that enables GPUs in computers to solve complex computing problems. It contains the CUDA instruction set architecture and the parallel computing engine inside the GPU, and the program can run with ultrahigh performance on the processor that supports CUDA.

The basic principle of CUDA is the idea of parallel computing, which decomposes a large computing task into several small computing tasks, so that multiple computing cores can be used to calculate these small tasks at the same time. When these small tasks are calculated, this large calculation task is also over. The CPU is designed to handle single or multiple tasks and is mainly used for serial computing, which is not effective in the face of a huge number of small computing tasks. GPU is composed of thousands of processors and is called streaming processors. The computing power of each processor core is not strong, but it performs well in the face of small tasks of parallel computing due to the huge number. The parallel computing of deep learning directly using CUDA is very complex. Therefore, the TensorFlow deep learning framework is used in this study. In TensorFlow, CUDA is written as a database that can be used directly in Python, bringing faster training speed and ease of use.

### 2.4. Human Exercise Intensity Recognition Method Based on ECG and PCG

The flow chart of this method is shown in Figure 3. Feature extraction and classification of ECG and PCG signals are performed using CNN, and exercise intensity detection is completed according to the classification results.

Step 1. First, collect the synchronized ECG and PCG signals in exercise, and then, process the ECG and PCG raw data to obtain a signal with denoised noise.

Step 2. In order to give full play to the feature extraction ability of the CNN network for two-dimensional images, we convert ECG and PCG into two-dimensional images, label the corresponding images, and divide the dataset of exercise intensity into training set and test set.

Step 3. Properly adjust the network structure parameters of AlexNet to adapt to the two-dimensional images of ECG and PCG signals, use the training set to train the AlexNet network, and use the test samples to test the training model. Finally, the exercise intensity classification model is obtained.

Step 4. Calculate the classification accuracy of exercise intensity on the test set, and output the classification result.

## 3. Dataset Processing

### 3.1. Introduction to the Dataset

This study uses the A Simultaneous Electrocardiogram and Phonocardiogram Database from the Physical Web for method validation [32, 33]. The study was approved by the Biomedical Engineering Review Committee (IRB equivalent) of Shiraz University, and the individuals gave written informed consent to participate in the study. A total number of 24 male subjects aged between 23 and 29 (average: 25.4 ± 1.9 years) participated in this study. Participants were in good physical condition, and no one shows or has ever experienced autonomic or cardiovascular disease symptoms as determined by structured interviews. The volunteers avoided food, caffeine, alcoholic beverages, and smoking for three hours before the test but were allowed to drink water regularly.

The resulting dataset consisted of 69 simultaneous ECG and PCG recordings, in which 8 records have a duration of 30 seconds and 61 records have a duration of 30 minutes. The resulting dataset was acquired simultaneously with a three-lead ECG and a single PCG stethoscope, sampled at 8 kHz, and the resolution is 12 bits. There are six different intensities of exercise, which are (1) laying on bed: the participants lie horizontally on the bed in a quiet room, and the ECG and PCG signals are recorded for 30 minutes at the same time; (2) sitting on armchair: ECG and PCG signals were recorded while the participant was sitting in the chair for 30 minutes; (3) walking at constant speed: the participants walked at a constant speed of 3.7 km/h for 30 minutes; (4) pedaling a stationary bicycle: participants ride on a stationary bicycle at a constant speed for 30 minutes; (5) on bicycle stress test: in the stress test, the load on the bicycle is continuously increased until it reaches excessive fatigue, excessive heart rate, or chest pain; and (6) on bruce protocol treadmill stress test: subjects run at a slower speed and then continuously increase the running speed until they reach excessive fatigue, excessive heart rate, or chest pain.

For the convenience of verification, only the first 6 modes are used for classification. As different exercise intensity simulations, the bicycle stress test and bruce protocol treadmill stress test are exercises in a dangerous state, and the experimenter will reach excessive fatigue, excessive heart rate, or chest pain. In these two states, the athlete should stop exercising. In order to be more specific, 6 different intensities of exercise are defined as 1-6 levels, and the exercise intensity increases with the level. When the exercise intensity is 5 or 6, the exerciser should stop exercising and have a rest. ECG and PCG signals are shown in Figure 4.

### 3.2. Divide Dataset

CNN have achieved great success in the field of image recognition. In order to make the data suitable for neural network training, one-dimensional ECG and PCG signal fusion is first required, and the fused data is converted into a two-dimensional image in a unified format. Such a method can maximize the preservation of the features contained in the one-dimensional signal.

The conversion method adopted in this study is to use the matplotlib plotting library in Python to convert the ECG and PCG into two-dimensional images. The first is to select an appropriate single sample length. The more data points a single sample contains, the richer the features it contains. However, if each sample contains too many data points, the total number of samples will be too small due to the limited data in the dataset, which is not conducive to the training of convolutional neural networks. By observing the laws of ECG and PCG signals, the signals show periodicity, and there are 6000-7000 data points between the peak and the peak of each cycle. So in order to ensure that each sample contains a complete cycle of ECG and PCG signals, select each sample to contain 10,000 data points. The divided 6 types of data are shown in Figure 5.

According to this method, ECG and PCG data are processed, and dataset 1 is obtained as shown in Table 1. The dataset is randomly divided into training set and verification set according to the ratio of 9 : 1.

The collection time of each athlete in the dataset is about 30 minutes, but the length of time is different. Under the condition of 8 kHz sampling, about 14,400,000 data points will be generated. Taking 10,000 data points as a sample, when the time is slightly more than 30 minutes, the number of samples generated by each athlete will be more than 1440, and when the time is slightly less than 30 minutes, the number of samples will be less than 1440. So, this will cause the number of samples in each category of the generated dataset to be different, which will also cause the data to be unbalanced during the training process. In order to balance the number of samples in each category of the dataset, data enhancement is performed on the data of the two categories of Exercise intensity 2 and Exercise intensity 6 to eliminate the data imbalance of the dataset. Since the original data is a one-dimensional sequence, we use a translation method to enhance the zoomed-in dataset, which is defined as multiscale clipping. Suppose *N* is the length of the original ECG time series dataset and *x* is the length of a data sample. After each sample is generated, the sample will be left some offset instead of being completely translated to the position of the next sample. According to the size of the offset, the multiple of data enhancement is determined. Dataset 2 as shown in Table 2 is obtained after data augmentation.

## 4. Experiments and Results

All experiments in this study were run on a Lenovo laptop with Windows 10 64-bit operating system, Intel® Core™ i7-10875H@2.30 GHz CPU, Nvidia GeForce RTX 2060 GPU, and 16 GB RAM. And data processing and enhancement were realized through Python. The CNN model is implemented using Python3.6 and the Keras deep learning library, and CUDA is used for accelerated computation during training.

### 4.1. Data 1: Imbalanced Dataset

The loss function curve and accuracy obtained from training Data 1 are shown in Figure 6. The final loss function value of the obtained model on the validation set is 0.2007, and the accuracy is 94.1%. This shows that the method of using ECG and PCG signal fusion to judge the exercise state is effective.

The confusion matrix puts the predicted results of all categories and the real results into the same table by category, in which there are the number of correct identifications and the number of incorrect identifications for each category. Cluster analysis of data can better observe the experimental results, find out the relationship between various categories, and make the data concise. The *t*-SNE technology can reduce the high-dimensional data of the fully connected layer of CNN to two-dimensional, so that we can visually and intuitively judge the performance of the current model. From this, the confusion matrix in Figure 7 and the cluster analysis in Figure 8 are obtained. Larger errors appear in category Exercise intensity 4. This may be because they are similar exercises and therefore have similar exercise intensities, therefore resulting in poor training results. This is the downside of using different datasets for validation.

### 4.2. Data 2: Balanced Dataset

The loss function curve and accuracy obtained from training Data 2 are shown in Figure 9. The final loss function value of the obtained model on the validation set is 0.1446, and the accuracy is 95.68%. This shows that the data imbalance does affect the training effect. By observing the resulting confusion matrix in Figure 10 and the cluster analysis in Figure 11, the number of Exercise intensity 4 which is identified as Exercise intensity 6 is reduced in the confusion matrix, and the change in the identification of Exercise intensity 3 is not obvious, which verifies the effectiveness of data augmentation for training. However, in order to further improve the accuracy, it is still necessary to collect different exercise intensities of a certain exercise in a targeted manner.

### 4.3. Comparison with Related Works

In this study, a deep learning approach was used to diagnose and classify the exercise intensity of athletes during exercise. To evaluate the classification performance of the proposed CNN model, we compared the accuracy of other methods for exercise intensity monitoring. In [34], they used data from a dual-axis accelerometer and a heart rate sensor, which is classified low, medium, and other forms of exercise; an accuracy of 84.65% was achieved. In [35], an analysis system constructed using CNN was used to evaluate the intensity and quality of exercise and obtained an accuracy of 93.5%. In [36], accelerometers placed at the joints were used to predict the intensity of physical activity and obtained experimental accuracies of 71.9-95.4% under different conditions. In [37], a health monitoring system based on wearable devices and smartphones was used to identify the intensity of activities, and a hierarchical algorithm composed of support vector machines (SVMs) had an identification accuracy of about 85%. In [38], they combined the Internet of Things (IoT), machine learning, and wearable technology to build a health and fitness analysis system that integrates data such as electrocardiogram, heart rate, heart rate variability, and respiratory rate, and the accuracy of identifying the physical state of athletes is able to reach 89%.

The comparison results are shown in Table 3 and Figure 12. The accuracy of the method in this study can reach 95.7%, and the prediction results of other research methods are 84.65%, 93.5%, 90.7%, 85%, and 89%, respectively, which demonstrates the effectiveness of the method proposed in this study. And most studies use data from well-designed laboratory settings for analysis, which has certain limitations. In the face of the real application environment, their generalization ability is poor and does not have the ability to customize. The method proposed in this paper uses neural networks and ECG and PCG signals to analyze exercise intensity. ECG and PCG signals are easy to obtain and have broad application prospects in practical applications.

## 5. Conclusion

In order to avoid the problems of physical damage caused by inappropriate exercise or training that cannot meet the actual needs, this paper proposes a method for human exercise intensity recognition based on ECG and PCG. We collect ECG and PCG signals from athletes with different exercise intensities, convert the signals into two-dimensional images, and send them to CNN for training. And then, this method is used to train and identify ECG and PCG signals in A Simultaneous Electrocardiogram and Phonocardiogram Database, the accuracy rate of 93.79% was obtained in the dataset without data enhancement, and the accuracy rate of 96.50% was obtained after data enhancement.

It can be seen from the training results that the use of ECG and PCG to identify exercise intensity has low complexity and is suitable for exercise intensity identification in various states, with strong robustness and effectiveness. Compared with the use of diagnostic methods with fewer features such as heart rate, it has broader application prospects. At present, the data used comes from the dataset collected by professional equipment, but this method has not been measured in actual sports, and the measurement accuracy of wearable acquisition equipment is also a major problem affecting the diagnosis effect during actual measurement. In future work, suitable wearable devices will be selected to collect ECG and PCG signals in a targeted manner to judge exercise intensity and to increase the diagnosis and prevention of diseases that may be caused by exercise.

## Figures and Tables

**Figure 1:** AlexNet network.

**Figure 2:** Confusion matrix.

**Figure 3:** Method flow chart.

**Figure 4:** ECG lead configuration and PCG stethoscope position for dataset.

**Figure 5:** Six different ECG and PCG fusion signals.

**Figure 6:** Loss and accuracy.

**Figure 7:** Data 1 confusion matrix.

**Figure 8:** Data 1 clustering analysis.

**Figure 9:** Data 2 loss and accuracy.

**Figure 10:** Data 2 confusion matrix.

**Figure 11:** Data 2 clustering analysis.

**Figure 12:** Comparison of accuracy of exercise intensity classification.

**Table 1:** Dataset 1.

Classes	Train set samples	Validation set samples
Bicycle	3877	430
Treadmill	2588	287
Stationary bicycle	3879	431
Walking at constant speed	3878	430
Laying on bed	3879	430
Sitting on armchair	2587	287

**Table 2:** Dataset 2.

Classes	Train set samples	Validation set samples
Exercise intensity 1	3879	430
Exercise intensity 2	3689	409
Exercise intensity 3	3878	430
Exercise intensity 4	3879	431
Exercise intensity 5	3877	430
Exercise intensity 6	3693	410

**Table 3:** Comparison of accuracy of exercise intensity classification.

Methods	Accuracy
Fernando et al.	84.65
Jian et al.	93.5%
Vahid et al.	90.7%
Igor et al.	85
Afzaal et al.	89
Proposed	95.7

## Data Availability

The adopted EEG dataset is acquired online, which is published by PhysioNet [32, 33]. Other data used to support the findings of this study are available from the authors upon request (wby1606443616@163.com).
